# Craniofacial similarity analysis through sparse principal component analysis

**DOI:** 10.1371/journal.pone.0179671

**Published:** 2017-06-22

**Authors:** Junli Zhao, Fuqing Duan, Zhenkuan Pan, Zhongke Wu, Jinhua Li, Qingqiong Deng, Xiaona Li, Mingquan Zhou

**Affiliations:** 1 School of Data Science and Software Engineering, Qingdao University, Qingdao, China; 2 College of Automation and Electrical Engineering, Qingdao University, Qingdao, China; 3 Engineering Research Center of Virtual Reality and Applications, Ministry of Education, Beijing, China; 4 College of Information Science and Technology, Beijing Normal University, Beijing, China; 5 College of Computer Science & Technology, Qingdao University, Qingdao, China; University College London, UNITED KINGDOM

## Abstract

The computer-aided craniofacial reconstruction (CFR) technique has been widely used in the fields of criminal investigation, archaeology, anthropology and cosmetic surgery. The evaluation of craniofacial reconstruction results is important for improving the effect of craniofacial reconstruction. Here, we used the sparse principal component analysis (SPCA) method to evaluate the similarity between two sets of craniofacial data. Compared with principal component analysis **(**PCA), SPCA can effectively reduce the dimensionality and simultaneously produce sparse principal components with sparse loadings, thus making it easy to explain the results. The experimental results indicated that the evaluation results of PCA and SPCA are consistent to a large extent. To compare the inconsistent results, we performed a subjective test, which indicated that the result of SPCA is superior to that of PCA. Most importantly, SPCA can not only compare the similarity of two craniofacial datasets but also locate regions of high similarity, which is important for improving the craniofacial reconstruction effect. In addition, the areas or features that are important for craniofacial similarity measurements can be determined from a large amount of data. We conclude that the craniofacial contour is the most important factor in craniofacial similarity evaluation. This conclusion is consistent with the conclusions of psychological experiments on face recognition and our subjective test. The results may provide important guidance for three- or two-dimensional face similarity evaluation, analysis and face recognition.

## Introduction

With the development of computer hardware and software, the computer-aided craniofacial reconstruction technique has become widely used in the fields of criminal investigation, archaeology, anthropology and cosmetic surgery. A similarity evaluation between the reconstructed face and the original face can be used to verify the effect of a craniofacial reconstruction, amend the reconstruction method and explore new reconstruction ideas. Craniofacial similarity analysis also has the following important benefits. In criminal investigations, it is helpful in assisting experts, witnesses and victims’ relatives in recognizing the faces of victims, to provide an identity and solve a criminal case more quickly. In the archaeological field, it has benefits in portraying ancient people with more realistic faces, improving the reconstruction results and providing an important reference value for archaeological research. In the medical cosmetic surgery field, it is useful for predicting the face remediation effect and providing reference data. It also has an important role in promoting the development of anthropology, in that anthropologists and biologists can learn about changes in the process of human growth and provide scientific support for the evolution of humans.

Reconstructed three-dimensional faces have their own characteristics and inaccuracies, owing to the use of different reconstruction techniques, and their similarity to the original faces directly reflects the pros and cons of the reconstruction methods used. The evaluation of craniofacial reconstruction results has become an important issue, and the current research work was motivated by the problematic paucity of research on the evaluation and analysis of reconstruction results.

The relevant research has focused on the field of the similarity of three-dimensional objects and face recognition. The study of three-dimensional object similarity has focused primarily on the comparison of two objects with entirely different shapes, which is relatively easy. However, the reconstructed craniofacial model and the original model are very similar in their overall shapes; therefore, many of the existing methods used for three-dimensional object similarity are not suitable, and the approaches appropriate for craniofacial similarity analysis are needed. Face recognition (FR) determines an identity on the basis of facial characteristics. The face features are usually extracted and used to recognize a face from a database, a given image or a video scene [1]. That is only to find the given face. In craniofacial similarity measurement, however, the main focus is on analysing whether an area is similar or dissimilar in shape, which is a more detailed and deeper question than in face recognition. Therefore, craniofacial similarity evaluation requires deep research.

In this paper, we propose the use of sparse PCA (SPCA) for 3D craniofacial similarity analysis, a method that can not only determine the similarity between two craniofacial models, but also identify regions of high similarity, which is important for improving the reconstruction effect. In addition, the areas that are important for craniofacial similarity analysis can be determined from the large amounts of data. This paper thus provides valuable information that may guide further studies.

## Related work

Craniofacial models belong to three-dimensional models. However, the methods of similarity evaluation of three-dimensional objects are mainly based on the geometry of an object, including its contour shape, topology shape and visual projection shape. Because the geometry of 3D faces is substantially identical, many of the similarity assessment methods for 3D objects are not applicable to evaluating 3D faces. To date, most scholars have evaluated craniofacial reconstruction results using subjective methods [2–7] to evaluate craniofacial similarity by collecting a certain number of tests and designing different evaluation strategies. Although this type of evaluation method is consistent with human cognitive theory, it requires a great deal of manpower and time, and the accuracy of the evaluation results is influenced by subjective human factors.

There are few objective evaluation methods for craniofacial reconstruction results. Some scholars have conducted preliminary explorations. Ip et al. [8] have presented a technique for 3D head model retrieval that combines a 3D shape representation scheme and hierarchical facial region similarity. The proposed shape similarity measure is based on comparing the 3D model shape signatures computed from the extended Gaussian images (EGI) of the polygon normal. First, the normal vector of each polygon of a head is mapped onto the Gaussian sphere, which is divided into cells, each of which corresponds to a range of orientations. Then, the cells are mapped onto a rectangular array to form a 1D shape signature. Finally, the total number of normal belonging to each cell on the rectangular array is counted, and the difference between any two signatures is revealed with a histogram. Wong et al. [9] have compared craniofacial geometries by taking the directions of the normal vectors as random variables and considering the statistical distribution of different cells as a probability density function. Feng et al. [10] have used a relative angle-context distribution (RACD) to compare two sets of craniofacial data. They defined the probability density function of the relative angle-context distribution and counted the number of relative angles in different intervals. To address the instability of calculation and long computing time problem of RACD, Zhu et al. [11] have extended the RACD to the radius-relative angle-context distribution (BRACD) algorithm by defining a set of concentric spherical shells and dividing the three-dimensional craniofacial points into different sphere ranges to calculate the relative angle in each partition for craniofacial similarity comparison. They have also proposed a method that uses the distances for different types of craniofacial feature points [12] and uses the principal warps method [13] to measure craniofacial similarity. Li et al[14] have put forward a similarity measure method based on iso-geodesic stripes. Zhao et al[15] have proposed a global and local evaluation method of craniofacial reconstruction based on a geodesic network. They defined the weighted average of the shape index value in a neighbourhood as the feature of one vertex and took the correlation coefficient’s absolute value of the features of all the corresponding geodesic network vertices between two models as their similarity. These methods are mainly analyses of craniofacial reconstruction results from the geometry.

Much research has focused on the field of face recognition, from 2D face recognition to 3D face recognition. Next, we provide a brief overview of 3D face recognition methods because they serve as a reference for craniofacial similarity evaluation.

### Feature-based methods

Feature-based methods recognize a face by extracting local or global features, such as curvature, curve, and depth value. Previous research on three-dimensional(3D) face recognition has focused mainly on curvature analysis. Lee and Milios[16], Gordon et al[17], and Tanaka et al.[18] have analysed the mean curvature and Gaussian curvature or principal curvature. Later, Nagamine et al.[19] proposed a method of matching face curves for 3D face recognition. Haar et al. [20] have computed the similarity of 3D faces by using a set of eight contour curves extracted according to the geodesic distance. Berretti et al. [21] have evaluated the similarity by using a three-dimensional model spatial distribution vector on equal-width iso-geodesic facial stripes. Lee et al. [22] have proposed a 3D face recognition method using multiple statistical features for the local depth information. Jahanbin et al.[23] have combined the depth of geodesic lines for identification. Recently Smeets et al. [24] have used meshSIFT features in 3D face recognition. Berretti et al.[25] have extracted the SIFT key points on the face scan and connected them into a contour for 3D face recognition. Drira et al. [26] and Kurtek et al. [27] have extracted the radial curves from facial surfaces and used elastic shape analysis for 3D face recognition. The face recognition efficiency of these methods is affected by the number or type of the characteristics extracted from the face.

### Spatial information methods

Spatial information methods directly match the surface similarity instead of extracting features, such as the Hausdorff distance method and iterative closest point (ICP) method. These methods are usually divided into two steps: alignment and similarity calculation. Achermann et al. [28] have used the Hausdorff distance to measure the similarity between point clouds of human faces. Pan et al. [29] have used a one-way partial Hausdorff as a similarity metric. Lee et al.[30] have used a depth value as a weight when using the Hausdorff distance for 3D face recognition. Chua et al.[31] have used ICP for three-dimensional face model precise alignment. Cook et al. [32] have established a corresponding relationship for a 3D face model by ICP. Medioni et al. [33] have performed 3D face recognition using iterative closest point (ICP) matching. Lu et al. [34] have proposed an improved ICP for matching rigid changing regions of a 3D human face and used the results as a first-class similarity measure. ICP is suitable for rigid surface transformation, but a face is essentially not a rigid surface, thus affecting the accuracy.

### Statistical methods

Statistical methods can obtain a general rule through applying statistical learning to many three-dimensional face models and then using these general rules for evaluation and analysis. Principal component analysis (PCA) has been used for face recognition. Vetter and Blanz[35] have utilized a 3D model based on PCA to address the problem of pose variation for 2D face recognition. Hesher et al.[36] have extended the PCA approach from an image into a range of images by using different numbers of eigenvectors and image sizes. This method provides the probe image with more chances to make a correct match. Chang et al. [37] have applied a PCA-based method using 3D and 2D images and combining the results by using a weighted sum of the distances from the individual 3D and 2D face spaces. Yuan[38] has used PCA to normalize both the 2D texture images and the 3D shape images extracted from 3D facial images and then recognized a face through fuzzy clustering and parallel neural networks. Theodoros et al[39] have evaluated 3D face recognition by using registration and PCA. First, the facial surface was cleaned and registered and then normalized to a standard template face. Then, a PCA model was created, and the dimensionality of the face space was reduced to calculate the facial similarity. Theodoros et al have used this technique on a 3D surface and texture data comprising 83 subjects, and the results demonstrate a wealth of 3D information on the face as well as the importance of standardization and noise elimination in the datasets. Russ et al. [40] have presented a 3D approach for recognizing faces through PCA, which addresses the issue of the proper 3D face alignment. Passalis et al [41] have used an annotated deformable model approach to evaluate 3D face recognition in the presence of facial expressions. First, they applied elastically adaptive deformable models to obtain parametric representations of the geometry of selected localized face areas. Then, they used wavelet analysis to extract a compact biometric signature to perform rapid comparisons on either a global or a per area basis.

Statistical methods are commonly used at present, but the classical method—PCA—cannot easily provide actual explanations. In this paper, we use the sparse principal component analysis (SPCA) method to evaluate craniofacial similarity, thereby effectively reducing the dimensionality and simultaneously producing sparse principal components with sparse loadings, and making it easy to explain the results. This methodology makes it possible to explain the similar and dissimilar parts between two craniofacial data and to carry out in-depth analysis. The SPCA method should therefore be more conducive to the evaluation of craniofacial reconstruction results.

## Materials and methods

### Materials

This research was carried out on a database of 208 whole-head CT scans on volunteers mostly belonging to the Han ethnic group in the North of China. The subjects’ ages ranged from 19 to 75 years, and 81 females and 127 males were included. The CT scans were obtained with a clinical multislice CT scanner system (Siemens Sensation16) in Xianyang Hospital located in western China. Our research was approved by the Institutional Review Board (IRB) of the Image Center for Brain Research, National Key Laboratory of Cognitive Neuroscience and Learning, Beijing Normal University. All participants gave written informed consent. The individuals in this manuscript have given written informed consent (as outlined in PLOS consent form) to publish these images.

First, we extracted the craniofacial borders from the original CT slice images (as shown in Fig 1A) and reconstructed the 3D craniofacial surfaces (as shown in Fig 1B) with a marching cubes algorithm [42]. After data processing[43], all 3D craniofacial data were transformed into a unified Frankfurt coordinate system[44][45] to eliminate the effects of data acquisition, posture, and scale. We selected a set of craniofacial data as a reference template and cut away the back part of the reference craniofacial model because there were too many vertices in the whole head, and the face features are mainly concentrated on the front part of the head. All of the craniofacial models were automatically registered with the reference model through the non-rigid data registration method [44], and each craniofacial data set (as shown in Fig 1C) had 40969 vertices.

**Fig 1:** The procedure of craniofacial data acquisition.

### Sparse principal component analysis (SPCA)

Sparse principal component analysis is a method developed from principal component analysis (PCA), which is a widely used technology for data dimensionality reduction. PCA seeks linear combinations of the original variables such that the derived variables capture the maximal variance.

**X** = (*x*_1_,*x*_2_,⋯,*x*_*p*_)′ is the set of original features, and **Y** = (*y*_1_,*y*_2_,⋯*y*_*p*_)′ is the set of new features that are linear combinations of the original features. PCA transforms the original vector by the equation Y = *T*'*X*, wherein the k-th principal component is

$${\text{y}}_{k}=t_{1k}x_{1}+t_{2k}x_{2}+\ldots +t_{pk}x_{p}$$ (1)

*t*_i*k*_ is called the **loading** of the k-th principal component y_*k*_ in the i-th original variable *x*_i_. The derived coordinate axes are the columns of T, called **loading vectors**, with individual elements known as loadings. Clearly, each principal component extracted by PCA is a linear combination of all of the original variables, and the loadings are typically non-zero. That is, the principal components are dependent on all of the original variables. This dependence makes interpretation difficult and is a major shortcoming of PCA. Therefore, we sought to improve PCA to make it easy to explain the results.

Hui Zou et al[46] have proposed sparse principal component analysis (SPCA) aiming at approximating the properties of regular PCA while keeping the number of non-zero loadings small. Sparse principal component analysis (SPCA) is an approach to obtain modified PCs with sparse loadings and is based on the ability of PCA to be written as a regression-type optimization problem, with the lasso[47] (elastic net[48]) directly integrated into the regression criterion, such that the resulting modified PCA produces sparse loadings. Next, we explain the lasso, the elastic net and the solution of SPCA.

#### Regression techniques

PCA can be written as a regression-type optimization problem, and the classic regression method is an ordinary least squares (OLS) approximation. The response variable *y*.is approximated by the predictors in X. The coefficients for each variable (column) of X are contained in *b* [49],

$$b_{OLS}=\text{arg}\;\underset{b}{\min}{\left|\left|y-Xb\right|\right|}^{2}$$ (2)

where ||·|| represents the L2-norm.

Hui Zou et al ^[^^46^^]^ have proposed obtaining sparse loadings by imposing the “elastic net” constraint on the regression coefficients. An L1-norm constraint, added on the basis of LASSO, can be written as

$$b_{nEN}=\text{arg}\;\underset{b}{\min}{\left|\left|y-Xb\right|\right|}^{2}+\lambda {\left|\left|b\right|\right|}^{2}+\delta {\left|\left|b\right|\right|}_{1}$$ (3)

where nEN is short for naive elastic net. The elastic net penalty is a convex combination of the ridge penalty and the lasso penalty, where *λ* > 0.

Next, we discuss how to calculate sparse principal components (PCs) on the basis of the above regression approach.

#### Sparse principal component analysis (SPCA)

Zou and Hastie have proposed a problem formulation called the SPCA criterion [46] to approximate the properties of PCA while keeping the loadings sparse.

(A^,B^)=argminA,B∑i=1n||xi−ABTxi||2+λ∑j=1k||bj||2+∑j=1kδj||bj||1SubjecttoATA=Ik (4)

The first part $\sum_{i=1}^{n}{\left|\left|x_{i}-AB^{T}x_{i}\right|\right|}^{2}$ measures the reconstruction error, and the other parts drive the columns of B towards sparsity, similarly to the elastic net regression constraints. The constraint weight *λ* has the same value for all PCs, and it must be chosen beforehand, whereas *δ* may be set to different values for each PC to offer good flexibility.

Zou and Hastie have also provided a reasonably efficient optimization method for minimizing the SPCA criterion in Ref [46]. First, if given A, Zou and Hastie has have proven that

$$\sum_{i=1}^{n}{\left|\left|x_{i}-AB^{T}x_{i}\right|\right|}^{2}+\lambda \sum_{j=1}^{k}{\left|\left|b_{j}\right|\right|}^{2}+\sum_{j=1}^{k}\delta_{j}{\left|\left|b_{j}\right|\right|}_{1}=TrX^{T}X+\sum_{j=1}^{k}(b_{j}^{T}(X^{T}X+\lambda )b_{j}-2a_{j}^{T}X^{T}Xb_{j}+\delta_{j}\;\left|\left|b_{j}\right|\right|)$$ (5)

This equation amounts to solving *k* independent naïve elastic net problems, one for each column of B.

Second, if B is fixed, A can be solved by singular value decomposition. If the SVD of B **is** B = UDV^T^, then A = UV^T^. Zou and Hastie [46] have suggested first initializing A to the loadings of the *k* first ordinary principal components and then alternately iterating until convergence because matrices A and B are unknown.

Thus, we can find the first *k* sparse components selected by the above SPCA criterion, and the detailed algorithm is provided in the next section. Then, the original data can be projected into the main direction to which the sparse principal components correspond. Thus, the dimensionality of the data is reduced.

### SPCA for craniofacial similarity measurement

Using SPCA for craniofacial similarity measurement, we first reduced every craniofacial datum’s dimensionality and projected them into the main-direction to which the sparse principal components corresponded to. Then, we computed the mean square error (MSE) between any two craniofacial data subjected to dimensionality reduction for comparison.

Before we evaluated the craniofacial similarity using SPCA, we ensured that all craniofacial data had a uniform coordinate system and had been registered. Then, the point cloud format data were used in the craniofacial similarity measure by SPCA. One point cloud format craniofacial datum was made by n (experimental data n = 40969) points, each containing three coordinates: *x*,*y*,*z*. To simplify the calculation, a craniofacial datum was converted to a one-dimensional vector including N(N = 3n) data. M craniofacial data (experimental data M = 108) were provided for the training sample set; i.e., a sample set was a N × M matrix, with each column denoting a craniofacial data set.

$$X_{j}^{T}=(x_{1j},x_{2j},x_{3j},\ldots x_{Nj})$$ (6)

We used 108 sets of point cloud format craniofacial data as training samples and then used the sparse principal component analysis (SPCA) method to find *k* sparse principal components. Then, we used 100 sets of point cloud format craniofacial data as test samples and projected them into a space of principal components. After *k* sparse principal components were selected by SPCA, the original data were projected into the main direction to which the sparse principal components corresponded for dimensional reduction. Then, we computed the mean square error of each pair of craniofacial data after the dimensionality reduction and determined the craniofacial similarity.

In the mean square error evaluation, we first compute the dimensional reduction vectors *y*_*i*_ and y_*j*_ through SPCA, which respectively are the projections in the main direction of craniofacial data vectors *x*_*i*_ and *x*_*j*_. Then we needed to determine the difference between two feature vectors *y*_*i*_ and y_*j*_ in different dimensions. We then calculated the square of the difference and averaged the results. The mean square error of the two craniofacial data was calculated with the formula

$$\text{s}(\text{i},j)=\frac{1}{L}\sum_{k=1}^{L}(y_{ik}-y_{jk}{)}^{2}$$ (7)

where *y*_*i*_ and y_*j*_ denote two craniofacial vectors subjected to dimensional reduction and *L* denotes the number of principal components. A smaller result of s(i,*j*) represents a smaller difference between the i-th craniofacial data and the j-th craniofacial data and a greater similarly degree.

On the basis of the above analysis, we constructed the algorithm for measuring craniofacial similarity by using SPCA as follows:

Input: Point cloud format craniofacial data
Output: Similarity matrix of every two craniofacial data
Step1: Read *M* sets of the point cloud format craniofacial data as training samples. The matrix X(N × M) is composed of *M* training samples, and each column datum of X is a craniofacial datum.
Step2: Find *L* sparse principal components and the primary directions by *M* training samples (craniofacial) using the SPCA method as follows.
  ① Let A start at V(1970), the loadings of first *k* ordinary principal components.
  ② Given a fixed A, solve the following naive elastic net problem for *j* = 1,2,…,*k*
    $$b_{j}=\arg\;\underset{b^{*}}{\min}b^{*T}(X^{T}X+\lambda )b^{*}-2a_{j}^{T}X^{T}Xb^{*}+\delta_{j}\;\left|\left|b^{*}\right|\right|$$
  ③ For each fixed B, do the SVD of X^T^XB = UDV^T^, and then update A = UV^T^.
  ④ Repeat steps 2–3, until B converges.
  ⑤ Normalization: ${\hat{V}}_{j}=\frac{b_{j}}{\left|b_{j}\right|}$, *j* = 1,2,…,*k*.
Step3: Read *T* sets of point cloud format craniofacial data as test samples and project them into the sparse primary directions to which the sparse principal components correspond. Calculate the new sample matrix after the dimensional reduction Y = V^T^X. In the same way, the original *N* dimensional data are reduced to the *L* dimension.
Step4: Compute the mean square error using formula (7) between two craniofacial data of *T* test samples after dimensionality reduction, and perform the similarity comparison and obtain a similarity matrix s.

### Analysis of the importance of each sparse principal component in craniofacial similarity comparison

Because the sparse principal components extracted by SPCA relate to only one or a few original variables, the results of the SPCA dimensional reduction can explain the meaning reflected by each principal component. V is the matrix of the extract sparse principal components, wherein each column is a sparse principal component vector, plus the mean face, and the expressed region of each sparse principal component can be seen. For example, one sparse principal component may reflect the area around the underjaw, and another may reflect the region around the mouth.

In the previous section, the craniofacial similarity measure was compared with all sparse principal components after dimensionality reduction; i.e., the similarity between the i-th craniofacial and the j-th craniofacial was calculated by the i-th row and the j-th row of the SPCA dimensionality reduction matrix Y according to the formula (7) (each row of Y represents a dimensionality reduction craniofacial data), and *L* is the total number of sparse principal components((in experiment *L* = 60). Therefore, we can calculate the proportion of sparse principal component *k* in the craniofacial similarity metric.

There are three calculations:

#### Calculate the proportion of each sparse principal component in all craniofacial comparisons

$$B_{k}=\frac{\sum_{i=1}^{\text{T}}\sum_{j=1}^{\text{T}}{\left(y_{ik}-y_{jk}\right)}^{2}}{\sum_{k=1}^{\text{L}}\sum_{i=1}^{\text{T}}\sum_{j=1}^{\text{T}}{\left(y_{ik}-y_{jk}\right)}^{2}}$$ (8)

B_k_ is the k-th sparse principal component proportion. In the above formula, each molecule denotes the sum of the similarity comparison values of the k-th sparse principal component when all T(T = 100) craniofacial data are compared. The denominator is the sum of the similarity comparison values of all sparse principal components (*L* is the total number of sparse principal components, in experiments L = 60 when all T(T = 100) craniofacial data are compared. The ratio is the proportion of the k-th sparse principal component in the comparison.

#### Calculate the proportion of each sparse principal component in the ten most similar craniofacial comparisons

The difference between this calculate and above calculate is that each molecule of this method calculates only the sum of the similarity comparison values of the k-th sparse principal component when each craniofacial datum is compared with the ten most similar craniofacial data. Thus, *L* is the total number of sparse principal components (in experiments L = 60), B_k_ is the proportion of the k-th the sparse primary component in the ten most similar craniofacial comparison.

$$B_{k}=\frac{\sum_{i=1}^{\text{T}}\sum_{j=1}^{10}{\left(y_{ik}-y_{jk}\right)}^{2}}{\sum_{k=1}^{\text{L}}\sum_{i=1}^{\text{T}}\sum_{j=1}^{\text{T}}{\left(y_{ik}-y_{jk}\right)}^{2}}$$ (9)

#### Calculate the proportion of each sparse principal component in the most similar craniofacial comparison

$$B_{k}=\frac{\sum_{i=1}^{\text{T}}{\left(y_{ik}-y_{1k}\right)}^{2}}{\sum_{k=1}^{\text{L}}\sum_{i=1}^{\text{T}}\sum_{j=1}^{\text{T}}{\left(y_{ik}-y_{jk}\right)}^{2}}$$ (10)

where *y*_1_ represents the highest similarity craniofacial data to the i-th craniofacial *y*_*i*_; i.e., the molecule calculates only the sum of the similarity comparison values of the k-th sparse principal component when each craniofacial data is compared with the most similar craniofacial data. Thus, *L* is the total number of sparse principal components (in experiments *L* = 60), B_k_ is the proportion of the k-th sparse principal component in the most similar craniofacial comparison.

After the proportions of each sparse principal component in the similarity comparison are calculated, the importance of each sparse principal component in the comparison results can be seen by sorting the proportions in descending order.

The detailed algorithm for calculating the sparse principal component in the comparison result according to importance is as follows:

① Read the craniofacial data of the point cloud format.
② Take *M* craniofacial data as training samples and obtain sparse principal components.
③ Derive the mean face by *M* craniofacial data.
④ Add each sparse principal component to the mean face and find the reflected area of each sparse principal component.
⑤ Calculate the proportions of each sparse principal component of craniofacial similarity measure in *T* test samples and sort them.

## Results

In our experiments, the preprocessed and registered craniofacial data (introduced in materials section) are used to compare the craniofacial similarity by PCA and SPCA method respectively. There 108 craniofacial data among the 208 CT scans were used as the training data and the other 100 skins were used as the test data for the craniofacial similarity comparison, i.e, M = 108 and T = 100 in our experiments. We use 108 craniofacial data to train the principal components by PCA and SPCA respectively, and use 100 craniofacial data to test their similarity. In SPCA method, the total number of sparse principal components L = 60 in our experiments. The experimental results are described as follows.

### PCA and SPCA similarity results comparison

#### PCA comparison results

We use the PCA and SPCA methods to reduce the dimensions of 100 craniofacial reconstruction data (test samples) and then used formula (7) to calculate the mean square error to compare the 100 craniofacial similarities. Finally, we obtained a similarity matrix s of 100 × 100. We took any ten similarity comparison results of PCA and produced the following Table 1:

**Table 1:** PCA results of the comparison (ten craniofacial data).

PCA	F1	F2	F3	F4	F5	F6	F7	F8	F9	F10
**F1**	0	6.3682	20.4600	13.6084	15.2861	5.4915	3.5066	134.5970	11.6981	8.7297
**F2**	6.3682	0	36.9393	17.9144	25.2519	4.1056	6.0655	165.2107	25.9621	9.0207
**F3**	20.4600	36.9393	0	18.0716	6.9442	22.7988	28.9824	65.6760	5.9180	29.5986
**F4**	13.6084	17.9144	18.0716	0	22.5093	6.2955	19.4578	92.3872	8.8958	5.9922
**F5**	15.2861	25.2519	6.9442	22.5093	0	17.5907	18.8078	87.8924	9.4349	24.2863
**F6**	5.4915	4.1056	22.7988	6.2955	17.5907	0	8.7473	121.1084	13.4716	4.3154
**F7**	3.5066	6.0655	28.9824	19.4578	18.8078	8.7473	0	159.8399	16.1770	9.2260
**F8**	134.5970	165.2107	65.6760	92.3872	87.8924	121.1084	159.8399	0	80.7340	131.0478
**F9**	11.6981	25.9621	5.9180	8.8958	9.4349	13.4716	16.1770	80.7340	0	13.4808
**F10**	8.7297	9.0207	29.5986	5.9922	24.2863	4.3154	9.2260	131.0478	13.4808	0

#### SPCA comparison results

We took the ten similarity comparison results of SPCA and produced the following Table 2:

**Table 2:** SPCA results of the comparison (ten craniofacial data).

SPCA	F1	F2	F3	F4	F5	F6	F7	F8	F9	F10
**F1**	0	0.4495	1.6585	1.1926	1.2289	0.4640	0.3544	10.8468	1.0918	0.7026
**F2**	0.4495	0	3.2704	1.5601	2.3552	0.3982	0.4776	13.5670	2.2592	0.7221
**F3**	1.6585	3.2704	0	1.6432	0.5779	2.1663	2.3313	5.5217	0.4337	2.3047
**F4**	1.1926	1.5601	1.6432	0	2.1196	0.6486	1.6096	7.9543	0.8496	0.4349
**F5**	1.2289	2.3552	0.5779	2.1196	0	1.7622	1.6348	7.0067	0.8953	2.2199
**F6**	0.4640	0.3982	2.1663	0.6486	1.7622	0	0.7595	10.0325	1.2963	0.4610
**F7**	0.3544	0.4776	2.3313	1.6096	1.6348	0.7595	0	13.0910	1.4565	0.8304
**F8**	10.8468	13.5670	5.5217	7.9543	7.0067	10.0325	13.0910	0	6.9895	10.8538
**F9**	1.0918	2.2592	0.4337	0.8496	0.8953	1.2963	1.4565	6.9895	0	1.2570
**F10**	0.7026	0.7221	2.3047	0.4349	2.2199	0.4610	0.8304	10.8538	1.2570	0

The top row and left-most column in the table refer to the numbers of the craniofacial models. The values of the i-th row and the j-th column sho w the mean square error between the i-th craniofacial and the j-th craniofacial. The smaller the mean square error is, the higher the similarity is. The diagonal elements are mean square error of each craniofacial against itself, which is 0, indicating complete similarity.

#### Comparison of SPCA and PCA results

In 100 craniofacial data, we used the PCA and SPCA methods to find the most similar data. The comparison indicated that in 100 sets of data, 35 (35%) sets of data were not identical, but the other 65 sets (65%) were the same in their ability to identify the most similar craniofacial data.

In our comparison of the different 35 sets of data results by SPCA and PCA methods (Fig 2), it can be seen from the following table that the SPCA results were significantly more similar to the target craniofacial model than were the PCA results.

**Fig 2:** Comparison of the closest craniofacial data found by SPCA and PCA.

We performed a test on the following 35 sets of data in which we randomly selected 50 testers to evaluate which one was most like the original craniofacial data in identifying the results of PCA and SPCA (in the test, the subjects did not whether the craniofacial data had been selected by PCA or SPCA). The test results showed that 92% of the testers (46 persons) thought that the craniofacial data selected by SPCA were more like the original data.

### Comparison of reflected area according to principal component in PCA and sparse principal component in SPCA

According to 108 sets of craniofacial data training sample, we calculated the mean face and then determined the principal components and sparse principal components by using the PCA and SPCA methods, respectively, and finally added the principal component of the PCA and sparse principal component of the SPCA to the mean face. The main area reflected by the principal component of PCA and sparse principal component of SPCA are shown in Fig 3 and Fig 4, respectively.

**Fig 3:** Reflected region by PCA principal component.

**Fig 4:** Reflected region by SPCA sparse principal component.

In the above figure, the blue area indicates that the results have the same value as the mean face; that is, there was no change in that region: the red area indicates the greatest change, and other coloured areas, such as yellow or green regions, indicate non-zero changes lower than those in the red areas. Thus, from Fig 3 and Fig 4, it can be seen that each PCA component reflects the whole or a larger region of a craniofacial, whereas each sparse SPCA component reflects only the local part of the craniofacial, such as the left figure mainly reflecting the head and nose area, the middle figure mainly reflecting the eye region and the right figure mainly reflecting the area of the mouth and chin. Therefore, the role of each of the sparse principal components of SPCA in the comparison of the craniofacial can be analysed.

### Importance analysis of each sparse principal component in the comparison of the results

PCA can be used to reduce the dimension and then compare craniofacial similarity. However, because the principal components extracted by PCA are associated with all of the original variables, it is difficult to use PCA to explain the results. SPCA effectively overcomes this defect in PCA. SPCA can not only reduce the dimension and calculates the craniofacial similarity, but also derive the contribution of each sparse principal component in the similarity measure. With formulas (8), (9), and (10), the proportion of each component was calculated to compare the similarity of the 100 craniofacial data. In accordance with the proportions arranged in descending order, we found the top ten important sparse principal components, and the results are shown in Fig 5, Fig 6 and Fig 7.

**Fig 5:** The proportion of each component in all craniofacial comparison.

**Fig 6:** The proportion of each component in the most ten similar craniofacial comparison.

**Fig 7:** The proportion of each component in the most similar craniofacial comparison.

The first row in the table indicates the importance ordering ID. The component in the front is more important than those in the back. The second line indicates the serial number of the sparse principal component, in order of importance. The third line reflects the corresponding area of the sparse principal component.

## Discussion

### PCA and SPCA similarity comparison results

The experimental results of PCA and SPCA similarity comparison indicated that in 100 craniofacial data, 65% of the results identifying the most similar craniofacial data by the SPCA and PCA methods were the same. When the comparison results were not the same, we performed a subjective test with 50 human subjects and concluded that 92% of the testers (46 persons) thought that the craniofacial selected by SPCA was more similar than that found by PCA. That is, on the whole, using the SPCA method to reduce the craniofacial data and perform similarity evaluation is better than using the PCA method.

According to the comparison of the reflected area by principal component in PCA and the sparse principal component in SPCA, each PCA component reflects the whole or a larger region of the craniofacial, whereas each sparse SPCA component reflects only a local part of the craniofacial, such as the mouth or nose. Thus, each sparse SPCA principal component reflects detailed areas. Hence, the sparse SPCA principal component, compared with the PCA principal component, can more easily explain the results.

### Areas with high similarity or dissimilarity in two craniofacial comparisons

By calculating the mean square error of each sparse SPCA principal component, we further analysed the areas with high similarity or dissimilarity of craniofacial, thus providing important guidance for improving the craniofacial reconstruction. If a sparse SPCA principal component has a small mean square error, it reflects an area with high similarity. In contrast, if a sparse SPCA principal component has a large mean square error, it reflects an area that is dissimilar.

For example, for craniofacial 2 (shown in Fig 8A), the most similar craniofacial found by the SPCA method was NO.53 (in the following Fig 8B). To the human eye, it is difficult to see the areas with high similarity. However, it can be seen that the following areas in the eye, mouth, and jaw are similar between them by comparing the first ten small MSE sparse principal components (as shown in Fig 9). Moreover, the following areas on the left and right sides of the face and the top of the head can be shown to be dissimilar by comparing the first ten large MSE sparse principal components (as shown in Fig 10). In Fig 8C, the regions with high similarity (blue area) and dissimilarity (e.g., red area, green area, yellow area) are visible on the whole.

**Fig 8:** The comparison of similar and dissimilar regions.

**Fig 9:** The regions with high similarity between F2 and F53 by SPCA sparse principal components.

**Fig 10:** The regions with dissimilarity between F2 and F53 by SPCA sparse principal components.

### The importance of each sparse principal component in the comparison results

From Figs 5–7, it can be seen that most of the first ten sparse principal components found by SPCA in the 100 test craniofacial data were associated with the face contour. For example, there were sparse principal components 3、2、10、8、4、5、and 33 in Fig 5; 3、2、10、6、8、5、and 4 in Fig 6; and 3、6、2、5、10、8、9、and 12 in Fig 7. Thus, there were 70% or 80% sparse principal components related to the face contours.

Because in the most similar craniofacial comparison, the proportion of the sparse principal component is more convincing, thus indicating that the face contours have the most important role in the craniofacial similarity measure. In addition, from Figs 5–7, we also conclude that the eyes and mouth have important roles in craniofacial similarity analysis.

These conclusions are consistent with the conclusions of psychology experiments on face recognition. The "face inversion experiment" in psychology research shows that global information is more often used when people recognize a face.[50] Generally speaking, the hair, facial contours, eyes and mouth are more important for face perception and memory. The craniofacial contour is the most important factor for craniofacial similarity evaluation in our experiment because our craniofacial data did not include hair.

These conclusions are also consistent with our subjective test. Of the fifty subjects, 57.78% thought that the craniofacial contour is most important for comparison, 26.66% thought that the eyes are the most important, 6.67% thought that the nose is the most important, 6.67% thought that the mouth is the most important, and 2.22% thought that other factors are the most important.

These results also reflect that the SPCA method can indeed identify the sparse principal components that play an important role in craniofacial similarity measures. Thus, the SPCA method can be used not only in craniofacial similarity analysis but also in other three- or two-dimensional face similarity measurements and analyses and in face identification.

## Conclusion

From the above discussion of the experimental results of craniofacial similarity analysis, it is clear that both PCA and SPCA can reduce dimension while maintaining the main features of the original data; thus, both processes can be used in craniofacial comparison. The results of these two methods are identical to a large extent. For inconsistent results, the SPCA results are superior to the PCA results. Most importantly, using SPCA in a similarity comparison allows not only comparison of the similarity degree of two craniofacial data but also identification of the areas of high similarity, which is important for improving the craniofacial reconstruction effect. The areas that are important for craniofacial similarity analysis can be determined from the large amounts of data. We conclude that the craniofacial contour was the most important factor for craniofacial similarity evaluation in our experimental data. These conclusions are consistent with the conclusions of psychology experiments on face recognition. Our results may provide important guidance in three- or two-dimensional face similarity evaluation and analysis and three- or two-dimensional face recognition.
